This article has been retracted.

# Mir-124 Attenuates STAT3-Mediated TH17 Differentiation in Colitis-Driven Colon Cancer

**DOI:** 10.3389/fonc.2020.570128

**Published:** 2020-12-17

**Authors:** Shiyong Lin, Qianwen Liu, Jing Wen, Kunhao Bai, Yandong Guo, Jing Wang

**Affiliations:** ^1^Department of Endoscopy, Sun Yat-sen University Cancer Center, State Key Laboratory of Oncology in South China, Collaborative Innovation Center for Cancer Medicine, Guangzhou, China; ^2^Department of Gastroenterology, Nanfang Hospital, Southern Medical University, Guangdong Provincial Key Laboratory of Gastroenterology, Institute of Gastroenterology of Guangdong Province, Guangzhou, China

**Keywords:** miR-124, STAT3, TH17 cell, colitis, colitis-related cancer

## Abstract

**Background:**

Inflammation often induces regeneration to repair the tissue damage. However, chronic inflammation can transform temporary hyperplasia into a fertile ground for tumorigenesis. Here, we demonstrate that the miR-124 acts as a safeguard to inhibit the pro-inflammatory production and reparative regeneration.

**Methods:**

The expression levels of miR-124 and IL-17, IFN-*γ* were detected by qRT-PCR. TH17 or TH1 cells were detected by flow cytometer, respectively. The binding of STAT3 to the promoter region of IL-17 gene was analyzed by Chip assay. miR-124 binding to the 3′UTR of STAT3 gene was detected by reported plasmid construction and luciferase assay. Furthermore, DSS-induced colitis mice model and T cell transfer model were used to confirm the function of miR-124 *in vivo*. The related gene expression was analyzed by ELISA and western blot experiments.

**Results:**

The results indicated that miR-124 decrease promotes colon tumorigenesis after *Citrobacter rodentium* infection and AOM/DSS induced colon cancer murine model. In molecular mechanism, miR-124 targets STAT3 to inhibit TH17 cell polarization and keep TH17 polarization in colonic microenvironment.

**Conclusions:**

Our study strengthened the important role of miR-124 in the regulation of adaptive immune responses and blocking the development of colitis-related cancer.

## Background

The development of colorectal cancer (CRC) is a process of host immune interaction between tumor and tumor microenvironment. Tumor cells secrete proinflammatory mediators, and immune cells secrete cytokines, which together can promote tumor process. Previous results have shown that the TH17 cells’ percent are higher in human CRC tissues (1, 2), which could activate immune suppressive mediators’ release, and weaken the activity of cytotoxic CD8^+^ cells to kill tumor cells (1, 3). TH17 cells are an important cytokines in various immune responses such as type 1 immunity, which produces IL-17 to be involved in adaptive immune response by IL-17/IL-17R signal pathway. Moreover, IL-17 also can accelerate neutrophil activation and coagulation. The previous studies confirmed that IL-17 expression step by step increased along with colonic adenomas to cancer process, but it is not a prominent mark to diagnose the CRC because IL-17 is not associated with TNM parameters of the tumor (4, 5). These results indicated that IL-17 oncogenous function might cooperate with other genes in colon cancer.

Many studies have demonstrated that MicroRNAs (miRs) are related to many human disease by cooperated with its target genes, such as colitis and colon cancer (6). Previous documents confirmed that miRs are involved in Toll-like receptor signaling, which is important to trigger the intestinal inflammation. For example, miR-146b induced by IL-10-IL-10R signaling regulated the Toll-like receptor 4 (TLR4) by negative feedback in human monocytes (7), and miR-146b deficient mice easily develop colitis by targeting IRF5 (8), which was regarded as a regulator of TLRs in LPS-driven TLR signaling. Moreover, strong pieces of evidence suggested that inflammation was the onset of cancer, and colitis also was closely related to colon cancer. However, it is still absent to explain relationships between colitis and colitis-related cancer (9). Many signaling pathway was involved in colitis-related cancer, including Toll-like receptors, PI3K/MAPK signaling, NF-*κ*B/STAT3 signaling, Wnt signaling, et al *(*10). In addition, more recent studies have indicated that miRNAs can target the above signaling molecules and connect inflammation to cancer development. Yuan et al. reviewed and listed that miRNAs were involved in inflammation to cancer. For example, miR-126 could directly target the CXCR4 or PI3K/AKT signaling pathway on tumor suppression (11, 12). Among those, miR-124 was down-regulated in pediatric UC patients, which targeted the STAT3 and increased the STAT3 expression. This data suggested that miR-124 epigenetically modified the pathogenesis coupled with its target genes in pediatric-UC (13). But, it is still unclear whether miR-124 can mediate the colitis-related cancer progression.

In current object, we demonstrated that miR-124 could inhibit the TH17 cell proliferation and was down-regulated in TH17 cell differentiation. The miR-124 mimic would retain in the inflamed area and efficiently inhibited the TH17 polarization, causing the phenotype transition into Treg cells, which next inhibited the inflammatory response and promoted the mucosal regeneration, and finally decreased the colitis-related colonic cancer development. Therefore, we expect targeting miR-124 would offer a novel therapeutic strategy for colitis-related colonic cancer.

## Methods and Materials

### Cell Line and Mice Model

The cell lines EL4, MC38, HEK293T were purchased from the American Type Culture Collection (ATCC) and cultured in RPMI-1640 (Invitrogen, CA, USA) with 10% fetal bovine serum (Gibco, CA, USA). C57BL/6J and Rag1^−−/−^ mice were obtained from Model Animal Research Center of Nanjing University and maintained in the barrier facility at Guangzhou Medical University. To construct the MC38 engrafts mice model, 5 × 10^5^ MC38 cells were injected subcutaneously into mice according to the document. The animal study protocols were approved by the Institutional Animal Care and Use by ethics committee of Sun Yat-sen University Cancer Center.

### Antibodies and Reagents

MiR-124 mimic were purchased from GenePharma. The following Flowcytometry antibodies were purchased from BD Biosciences (USA), such as FITC-CD4 (L3T4, 553729), APC-CD25 (PC61.5, 557192), PE-IL-17 (TC11-18H10, 559502), PE-cy7-IFN-*γ* (XMG1.2, 561040), PE-FOXP3 (FJK-16S, 560408) and isotype controls. Antibodies for ROR*γ* (562197) were purchased from BD Bioscience. FITC Annexin V Apoptosis DetectionKit I (2293683) was purchased from BD Pharmingen. anti-T-bet (Invitrogen,14-5825-82), anti-STAT3(cell signaling technology, 4368), anti-pSTAT3 (Cell Signaling Technology, 4074), ago2 antibody (proteintech, 10686-1-AP), and anti*-β*-actin (Sigma, A5441) antibodies for western blotting were used according to the manufacturers’ instructions. Secondary antibodies were from Santa Cruz Biotechnology, Inc.

### CD4^+^ T Cell Preparation and Differentiation *In Vitro*

Naive CD4^+^ T cells were isolated by magnet sorting system from spleens and lymph nodes of C57BL/6 mice according to previous description (14). The sorted cells were primed for 96 h with anti-CD3 (1 μg/ml; 145-2C11; BD Biosciences) and soluble anti-CD28 (2 μg/ml; 566883; BD Biosciences). Cells stimulated under neutral conditions were defined as TH0 cells. Cells were stimulated to differentiate into TH1 cells by supplementation with IL-12 plus anti-IL-4 or into TH2 cells by supplementation with IL-4 and anti-IFN-*γ*. For TH17 cell differentiation, cells were stimulated with transforming growth factor-*β*1 (5 ng/ml, 7346-B2/CF), IL-6 (20 ng/ml, P08505) and IL-23 (10 ng/ml; 1887-ML, all from R&D Systems) and into Treg cells by supplementation with transforming growth factor-*β*1 (15 ng/ml).

### Intracellular Staining, ELISA Detection

For CD4^+^ cells staining, CD4^+^ cells were stimulated with PMA andionomycin for 5 h in the presence of brefeldin A prior to intracellular staining, and fixed with IC Fixation Buffer according to the manufacturer’s instructions (BD Bioscience, 554714). After staining the antibodies, cells were detected by FACS Calibur (BD Biosciences). Cell cultured supernatants were collected and detected by different ELISA Kits according to the manufacturer’s instructions and according previous description (8).

### RNA Isolation and Quantitative Real-Time RT-PCR

Total RNA was extracted using an RNeasy pluskit (QIAGEN, 74136, Valencia, CA), and cDNA was generated with an oligo (dT) primer and the Superscript II system (Invitrogen, 18064022, USA) followed by analysis using iCycler PCR with SYBR Green PCR master Mix (Applied Biosystems, 4309155). Results were normalized based on the expression of actin. IL-17 primer: Forward: 5′-CTCCAGAAGGCCCTCAGACTAC-3′, Reverse: 5′-AGCTTTCCCTCCGCATTGACACAG-3′, IFN-*γ* primer: Forward: 5′-ACTGGCAAAAGGATGGTG-3′, Reverse: 5′-GTTGCTGATGGCCTGATT-3′. *β*-actin: Forward: CATTGCTGACAGGATGCAGAAGG, Reverse: TGCTGGAAGGTGGACAGTGAGG.

### Luciferase Activity Assay

The sequence of stat3 3′UTR binding to miR-124 was cloned into the pMIR-REPORT™ miRNA Expression Reporter Vector System (Thermo Fisher, AM5795) according to instruction with the restrict enzyme HindIII and Spel. Stat3 primers: forward: 5′-CCCAAGCTTGGGTCAACCTGCCTTCCTTTCCC-3′ and reverse: 5′-GGACTAGTCC GGCAATCCCTCTCGACACAA-3′. Stat3 mutant primers: forward: 5′-CCCAAGCTTGGG ATGTCCAAAGGCCCTCTGTC-3′ and reverse: 5′-GGACTAGTCC GGCAATCCCTCTCGACACAA-3′. The cells were transiently cotransfected in 96-well plates with a luciferase reporter vector containing 3′-UTR wild or variants plasmid with miR-124 mimic as described. After 48 h, luciferase activity was measured with Dual-Glo Luciferase Assay System (E2920, Promega, WI, USA), and Renilla luciferase activity was normalized to Firefly luciferase activity.

### Western Blot

Equal amounts of protein samples were run on a 10% SDS-PAGE gel and blotted onto a polyvinylidene difluoride membrane [Bio-Rad]. Protein blots were incubated with the primary antibody at 4°C overnight and then with the appropriate secondary antibody for 1–2 h at room temperature, followed by detection with an enhanced chemiluminescence detection system.

### RNA Immunoprecipitation and Chromatin Immunoprecipitation Assay

RIP assay was performed as previously described (8). Briefly, an aliquot of immunoprecipitation supernatants, corresponding to 1 × 10^6^ cell equivalent, was removed after immunoprecipitation as “input”. Results were expressed as fold enrichment relative to Ago2-immunoprecipitation control samples. For Chip assay, ChIP was performed using an assay kit following the manufacturer’s instruction (Thermo Fisher, 26162), and briefly, ELF4 cells after the treatment of control or miR-124 mimic were cross-linked by exposure to 1% formaldehyde for 10 min at 37°C. Nuclei were prepared and subjected to sonication to obtain DNA fragments. Anti-STAT3 antibody was employed to pull down the DNA fraction after protein A-agarose beads preclearing. The input and immunoprecipitated DNA were amplified by qPCR using primers encompassing the known STAT3 binding sites on the IL-17 promoter region according to previous document (8).

### CD4^+^ T Cell-Transfer Colitis Model

T cell transfer colitis was performed as previously described. Briefly, purified CD4^+^ T cells from WT mice were injected intraperitoneally into Rag1^−/−^ recipients (5 × 10^5^ cells per mouse in 200 μl sterile PBS per injection) (15). Mice weights were recorded every week in whole experiments. The degree of inflammation in the epithelium, submucosa, submuscularis propria, and colitis scoring was elevated as described previously (8).

### Histochemistry, Immunohistochemistry, and Immunofluorescence

According to previous description (16), briefly, the H&E and immunohistochemistry were independently performed and histological scoring of inflammation and identification of tumors were evaluated by two senior pathologists referring to published document (8).

### AOM/DSS Mouse Model

We constructed the colitis-associated colorectal carcinoma by AOM/DSS administration according to document (16). Mice were intraperitoneally injected with 10 mg/kg body weight azoxymethane [AOM, 25843-45,Sigma-Aldrich Corp.DSS, 9011-18-1, molecular weight 36,000–50,000 Da, MP Biomedicals, USA]. One week later, mice were given 3% DSS in distilled water for 7 days followed by 14 days of normal drinking water as previously described. This cycle was repeated three times. Mice were sacrificed after the third cycle ended.

### *C. rodentium* Infection Colitis Colon Cancer Murine Model

*C. rodentium* Strain DBS100 was purchased from ATCC and cultured according to published methods (17, 18). 2 × 10^9^ CFU *C. rodentium* were infected into 8 weeks old mice by oral gavage. After six months, all mice were sacrificed and tumor occurrence was detected

### Statistical Analysis

The results are shown as means ± SD and statistical analysis was performed using Student’s t-test. Where more than two groups were compared, one way-ANOVA with Bonferroni’s correction was performed. P <0.05 was considered statistically significant.

## Results

### MiR-124 Inhibited the TH17 Cell Polarization

In order to study the effect of miR-124 on the function of adaptive immune cells, we first focused on T helper cells. Purified CD4^+^ T cells from C57BL/6 mice were subjected to primer *in vitro* for 3 days under TH0, TH17, Treg and TH1 conditions, and the expression of miR-124 was evaluated by qPCR. We found that miR-124 expression was significantly reduced in TH17 cells but not in TH1 (**Figure 1A**). qPCR and ELISA experiments showed that miR-124 mimics significantly inhibited the expression of TH17 or TH1 related genes (including IL-17, IFN-*γ*) (**Figures 1B–E**). Next, we tested whether the differentiation of TH17 and TH1 cells was affected in the presence of miR-124 mimics. These observations were related to the reduction in IL-17 and IFN-*γ* production by flow cytometry in TH17 or TH1 cells treated with miR-124 mimics (**Figure 1F**). The results showed that IL-17 and IFN-*γ* production were reduced after the treatment of miR-124 mimics. In order to exclude the possibility that the abnormal cells apoptosis was caused by miR-124 mimic, we isolated and analyzed CD4^+^ T cells from spleens as well as lymph nodes of C57BL/6 mice by Annexin V and PI staining or CSFE staining. The results showed that miR-124 mimic administration did not increase the T cell apoptosis but affected the CD4^+^ cell proliferation (**Figures 1G, H**).

**Figure 1:** miR-124 selectively suppresses TH17 and T_H_1 cell differentiation. **(A)** miR-124 expression in TH0, TH17, TH1, and Treg polarizing conditions by qPCR assay. Naïve CD4^+^ T cells from C57BL/6 mice were differentiated under TH17 and TH1 polarizing conditions respectively in the presence of 4.8 nmol miR-124 mimic for 3 days and analyzed through qPCR assay **(B, C)**. ELISA **(D, E)**, and flow cytometry **(F)**. **(G)** Naïve CD4^+^ T cells from C57BL/6 mice were differentiated under TH17 polarizing conditions respectively in the presence of 4.8 nmol miR-124 mimic for 3 days and analyzed through flow cytometry. **(H)** CD4^+^ cell proliferation was detected by CSFE. **(G)** Naïve CD4^+^ T cells from C57BL/6 mice were differentiated under TH17 polarizing conditions respectively in the presence of 4.8 nmol miR-124 mimic for 3 days, and stained with Annexin-V, analyzed through flow cytometry. *p < 0.05, **p < 0.01 *versus* cells cultured. All tests were performed three times.

#### MiR-124 Altered the Binding Activity of STAT3 to IL-17 Promoter in TH17 Cells

In addition, we explore the molecular basis of how miR-124 regulated TH17 cell differentiation. Since many studies have shown that multiple transcription factors including ROR*γ*t, STAT3, and AHR were important for the differentiation of TH17 cells, we suspected that miR-124 might affect the expression of these transcription factors. To solve this problem, naive CD4^+^ T cells from C57BL/6 mice were primed *in vitro* for 3 days under TH0 or TH17 transformation conditions. In the presence of miR-124 mimics, IL-17 mRNA was detected and the results showed that miR-124 mimics can inhibit IL-17 expression (**Figure 2A**). However, the levels of ROR*γ*t and AHR proteins were comparable in the presence of miR-124 mimics (**Figure 2B**), but STAT3 expression decreased after miR-124 mimics’ treatment (**Figure 2C**). ChIP analysis showed that the binding of STAT3 to the IL-17 gene promoter region was significantly reduced (**Figure 2D**). The data showed that miR-124 could inhibit the expression of STAT3 under TH17 cell differentiation conditions and then affected the expression of IL-17.

**Figure 2:** miR-124 suppresses TH17 activation by targeting STAT3. Naïve CD4^+^ T cells from C57BL/6 mice were differentiated under TH17 and TH1 polarizing conditions with IL-6 (10 ng/ml) and TGFβ (5 ng/ml) for 24 or 72 h in the presence of 4.8 nmol miR-124 mimic. **(A)**, miR-124 expression was detected by qPCR, U6 as control. **(B, C)** The whole cell lysates were prepared, and western blotting was performed for the analysis of protein expression. B-actin expression serves as a control. **(D)** El4 cell was stimulated with CD3 and CD28 antibody and primed with IL-6 and TGFβ in the presence of miR-124 mimic. Chip assay was performed with anti-STAT3 antibody, IgG antibody as negative control. *p < 0.05; **p < 0.05, miR-124 mimic vs Control in the present of IL-6/TGFβ. The results are representative of three independent experiments.

#### miR-124 Targeted on STAT3 in TH17 Differentiation

We further investigated how miR-124 affects the STAT3 in TH17 cell differentiation. The previous document and biomat information analysis revealed that miR-124 could bind the 3′UTR of STAT3 gene and inhibit the protein translation (13). To verify that miR-124 really targets STAT3, we first detected that STAT3 was affected in the presence of miR-124 mimic, and the results suggested that miR-124 mimic decreased the STAT3 expression in EL4 cell line (**Figure 3A**). Next, we constructed the luciferase reporter plasmids of the STAT3 3′UTR of mouse (including WT and miR-124 bind site mutant plasmids). miR-124 mimics were respectively co-transfected with the plasmids to El4 or HEK293T cells. The data suggested that miR-124 mimic significantly suppressed the luciferase activity in the STAT3 plasmid group. Collectively, the data also confirmed that miR-124 mimic had no effect on luciferase activity in the STAT3 mutant plasmid group (**Figures 3B–D**). Furthermore, we performed RNA immunoprecipitation (RIP) experiments to verify that both miR-124 and STAT3 mRNA were located at the same miRNA-induced silencing complex (miRISC) (**Figure 3E**). Taken together, the results suggest miR-124 modulates TH17 differentiation by targeting STAT3.

**Figure 3:** STAT3 is the target of miR-124. **(A)** EL4 cells were primed with IL-6 and TGFb in the presence of miR-124 mimic. STAT3 protein level was evaluated by western blotting. **(B)** Schematic representation of wild-type (wt) and mutant (mut) STAT3 3′UTR luciferase reporter constructs of predicted miR-124 target gene. The miR-124 binding region is indicated. **(C)** EL4 cells were co-transfected with miR-124 mimic and STAT3 3′UTR luciferase reporter plasmid after priming with IL-6 and TGFβ. **(D)** 293 T cells were co-transfected with either WT or mutant STAT3 luciferase reporter plasmids together the miR-124 mimic for 48 h. The cell lysates were prepared and luciferase activity was determined (Data represent mean ± s.d.). **(E)** EL4 cells were primed with IL-6 and TGFb in the presence of miR-124 mimic for 24 h. Total RNA was extracted and immunoprecipitated with anti-Ago2 antibody. The immunoprecipitated RNA was purified, and qPCR was performed for the analysis of miR-124 and STAT3 mRNA expression (Data represent mean ± s.d.). The results are representative of three independent experiments (Data represent mean ± s.d.). The results are representative of two independent experiments. *p < 0.05, **p < 0.01; ns indictated the negative significance.

#### MiR-124 Weakened the Colitis in a CD4^+^ Cells Transfer Model

To further evaluate the effect of miR-124 on the development of TH17 cells *in vivo*, we used CD4^+^ cells from C57BL/6 mice to induce Rag1−/− mouse colitis. The mice in the treatment group received low-dose miR-124 mimic twice a week for 8 weeks while control group was treated with PBS. Rag1−/− mice recombined with pure CD4^+^ T cells continued to lose weight, but treatment with miR-124 mimic can significantly improve their condition (**Figures 4A, B**). A parallel histological study of colon sections of Rag1−/− mice treated with miR-124 mimic showed that the pathological score was significantly increased compared with mice treated with PBS (**Figure 4C**). In addition, miR-124 expression was also confirmed in the treatment of miR-124 mimics (**Figure 4D**). Compared with the PBS-treated mice, the proportion of IL-17 cells in mice treated with miR-124 mimic was significantly reduced, and TH17, TH1 signature genes are also decreased (**Figures 4E, F**).

**Figure 4:** MiR-124 weakened the colitis in CD4 positive cell transfer model *in vivo*. CD4^+^CD45Rb^hi^ T cells were purified from C57BL/6mice and 5 × 10^5^cells were injected (i.p.) into recipient *Rag1*^−/−^mice. Mice were treated with control or miR-124 mimic (at 10 nm/mouse) every three days. **(A)** Morphology of intestines; **(B)** disease scores, *p < 0.05 *versus* recipients of control group (*n* = 5–6 mice per group); **(C)** sections of colons with colitis from *Rag1*^−/−^ mice (*n* = 5–6 mice in each group) 8 weeks after naïve T cell transfer as described above. Scale bar, 100 μM. **(D, E, F)** The percentage of IL-17 -producing cells from mesenteric lymph nodes and LPL of *Rag1*−^/^− mice in control and miR-124 mimic treated group. ***p < 0.001 *versus* recipients of control treated group.

### MiR-124 Suppressed the Development of Colitis Associated Carcinoma by Inhibiting the TH17 Differentiation

Ulcerative colitis (UC) was easier to develop into colon cancer, which included two important pathophysiological features: dysregulation of immune system and impaired mucosal repair. As previously reported, TH17 cell differentiation was closely related to CRC occurrence. After constructing the CRC mice model with DSS-Water return feed, the data showed that miR-124 mimic treatment group developed significantly smaller tumor numbers and tumor areas than the controlled group (**Figure 5A, B**). In addition, histological evaluation revealed that mice colonic mucosa after miR-124 mimic treatment showed low-grade dysplasia, while other tumors were usually identified as high-grade dysplasia (**Figure 5C**).

**Figure 5:** miR-124 suppressed the development of colitis associated carcinoma by inhibiting the TH17 differentiation. **(A)** Schematic of AOM/DSS administration. Mice were injected with 12.5 mg/kg AOM and subjected to three 7-day cycles of 2.5% DSS respectively in the presence of control or miR-124 mimic. **(B, C)** Morphology of intestines and representative H&E-stained sections and PAS after DSS or AOM/DSS treatment. Scale bar: 100 μm. **(D)** Total RNA was extracted and mRNA was detected by qPCR, b-actin as control. *P < 0.05; **P < 0.01. The results are representative of three independent experiments. **(E)** The percentage of IL-17-producing cells from mesenteric lymph nodes of mice in control and miR-124 mimic treated group. *p < 0.05 *versus* recipients of control treated group.

Moreover, for acute mucosal injury, miR-124 mimic promoted the better epithelium structures concomitant with the lower expression of IL-17. In the process of the CRC, IL-17 expression in miR-124 mimic treated mice was lower than that in the controlled group (**Figures 5D, E**), suggesting that chronic inflammation by AOM/DSS impaired the colonic epithelial microenvironment and the TH17 cells function, resulting in development of inflammation induced cancer, and TH17 cells were recruited around the neoplastic epithelial cells in regeneration, and the concomitant alteration was also exhibited in stat3 expression. Therefore, miR-124 disturbed the process of CRC by attenuating the inflammation before carcinogenesis

### MiR-124 Depressed the Colon Carcinogenesis in *C. rodentium* Infection Colitis Colon Cancer Murine Model

Microbial dysbiosis causes chronic inflammation associated with CRC. *C. rodentium* is a mucosal pathogen of mice and has a common pathogenic mechanism and 67% of genes with pathogenic colon (EPH) and enterohemorrhagic *Escherichia coli* (EHEC) *in vivo*, which are two important human gastrointestinal pathogens. *C. rodentium* implants have been used as models for studying mucosal immunology, including bacterial-induced colitis and parasitic reactions during the development of colon tumors.

After *C. rodentium* (2 × 10^9^ CFU) infection, WT mice developed diarrhea and weight loss within 2 weeks and were then divided into two groups: miR control and miR-124 mimic. Until 6 months, all mice were sacrificed and we performed histologic staining analysis. Microscopic sections from WT control mice were not mucosal dysplastic and neoplastic changes at six-month time points infection. In miR-124 mimic treatment mice, less dysplasia or early neoplasia was present at this time point, whereas 16/20 (WT control) *vs* 5/20 (miR-124 mimic) mice had microscopic changes ranging from dysplasia to adenocarcinoma (**Figures 6A, B**). We further isolated CD4^+^ T cells from *C. rodentium*-infected colon cancer tissue and analyzed the percent of TH17 cells and the IL-17 expression. IL-17 was significantly decreased after miR-124 treatment (**Figures 6C, D**). So, miR-124 mimic treatment expressed the TH17 cell differentiation in the colon post *C. rodentium* infection.

**Figure 6:** MiR-124 depressed the colon carcinogenesis in C. *rodentium* infection colitis-related cancer murine model. 8-week-old wild-type mice (WT; n = 12) infected orally with 2 × 10^9^ colony-forming units (CFUs) of C. *rodentium* in the presence of control (n = 6) or miR-124 mimic (n = 6). **(A, B)** Morphology of intestines and representative H&E-stained sections and PAS after C. *rodentium* infection. Scale bar: 100 μm. **p < 0.01 versus recipients of miR-124 mimic treatment group. **(C)** Total RNA was extracted and mRNA was detected by qPCR, b-actin as control, *P < 0.05; **(D)** The percentage of IL-17-producing cells from mesenteric lymph nodes of mice in control and miR-124 mimic treated group. *p < 0.05 *versus* recipients of control treated group.

## Discussion

Limited therapies available at present remains a challenging problem for the clinician in UC and colitis-related colon cancer. In our study, we confirmed the miR-124 was a key regulator for TH17 cell differentiation in UC and CRC, and performed the miR-124 mimic to effectively inhibit the colitis and colon cancer occurrence in murine colitis model. Thus miR-124 could block TH17 cell differentiation and pro-inflammatory cytokine induction and strengthen the mucosal repair, which suppressed the development of colitis associated carcinoma. We concluded that miR-124 is a critical regulator in control of intestinal immune function and epithelial regeneration, and targeting miR-124 can be selected as a “smart” therapeutic strategy for UC and colitis-related colon cancer.

The host immune system always combated with mutant cells during CRC development, which decided the good or malignant outcome (19). IL-17 is a pro-inflammatory cytokine, which is associated with many cancer progressions, which is mostly derived of T-helper17 (TH17) cells (20, 21) In colon cancer, published document showed that TH17 was involved in colitis and colitis-related cancer and also could mediate the activity of CTLs in colon cancer development (3, 22). Although the physiological level of inflammation was protective, excessive inflammation was harmful and the basis of inflammatory bowel disease (IBD) and inflammation-promoted colorectal cancer. Cytokine and transforming and degrading enzymes, growth factors, and reactive oxygen species together promoted tumorigenesis. A microenvironment was beneficial to intestinal epithelial cell proliferation, cell survival, and invasiveness. In our study, TH17 also was verified to be related with colon cancer development. But how to regulate the TH17 cell differentiation still was elusive.

RORγ, AHR and STAT3 are the transcription factors responsible for TH17 differentiation and stabilization. Gerogios et al. demonstrated that miR-124 could promote the children UC and pathogenesis by regulating the expression and phosphorylation of STAT3, but special cell type was not involved (13). The previous study also demonstrated that miR-124 depression was related to carcinogenesis and development by targeting different genes (23–25). These observations suggested that miR-124 played a key role in colitis and sporadic colon cancer. In our present study, we focused on the miR-124 function in TH17 cell and found that miR-124 could inhibit the polarization of TH17 cell and promote the transition of TH17 to treg in colitis and colitis-related colon cancer by targeting stat3 gene. Strangely, the ROR*γ* and AHR expression showed little change after the treatment of miR-124 mimic (**Figure 2B**). This change was also exhibited in a previous document, and authors explained that the epigenetic modification of STAT3 promoted the earlier TH17 cell differentiation regardless of ROR*γ*t and other IL-17 related transcription factors (26, 27). Moreover, these results also are consistent with down-regulation of miR-124 developing intestinal failure with M1 macrophage phenotype by targeting stat3 and acetylcholinesterase (AChE). We believe that in the absence of miR-124 signaling cascade, the presence of intestinal commensal bacteria will drive intestinal CD4^+^ T helper cells toward TH17 cell polarization, resulting in a hyper-inflammatory response with associated tissue damage and pathogenesis.

Collectively, our results confirmed that miR-124 expressed in TH17 cell shaping of TH17 polarization. The data suggested that a novel mechanism for the effect of miR-124 targeting STAT3 in the modulation of TH17 cell differentiation. miR-124 mimic obviously suppressed TH17 cell differentiation by inhibiting STAT3 level and IL-17 related genes *in vitro* and ameliorated colitis and CRC development *in vivo*. So, the results show that miR-124 acts as a key role in the modulation of TH17 cell activation and strengthens the potential role of miR-124 in the control of immune responses and pathogenesis of inflammatory diseases. And it was important that miR-124 mimic suppressed the TH17 differentiation during colitis process and delayed or inhibited the development of colitis-related cancer. The previous document suggested that blocking colitis could effectively decrease the occurrence of CRC (18). Further, our findings from mouse models suggested an application that miR-124 could serve as a biologic therapy in ameliorating colitis and CRC.

## Data Availability Statement

The raw data supporting the conclusions of this article will be made available by the authors, without undue reservation.

## Ethics Statement

The animal study was reviewed and approved by Institutional Animal Care and Use Committee of Sun Yat-sen University Cancer Center.

## Author Contributions

Conceptualization and methodology: SL and JWa. Formal analysis and data collection: JWe, YG, and KB. Writing—original draft preparation and Writing—review and editing: SL and JWa. All authors contributed to the article and approved the submitted version.

## Funding

This work was in part supported by Open Project Fund of Guangdong Provincial Key Laboratory of Gastroenterology (2017), and Foundation of President of Nanfang Hospital (2016Z015).

## Conflict of Interest

The authors declare that the research was conducted in the absence of any commercial or financial relationships that could be construed as a potential conflict of interest.

## Abbreviations

CRC, Colitis-Related Cancer; miR-124, microRNA-124; qPCR, quantitative real-time PCR; DSS, Dextran Sulfate sodium salt; AOM, azoxymethane.
